The article "Genetic Testing for Successful Cancer Treatment" was retracted in 2025. Reason: concerns about the authorship.

# Genetic Testing for Successful Cancer Treatment

**DOI:** 10.7759/cureus.49889

**Published:** 2023-12-04

**Authors:** Desh Nidhi Singh, Sushma Daripelli, Mohamed Osman Elamin Bushara, Georgiy Georgievich Polevoy, Muthu Prasanna

**Affiliations:** 1 Microbiology, Rama Medical College Hospital & Research Centre, Kanpur, IND; 2 Anatomy, Government Medical College (GMC) Jangaon, Jangaon, IND; 3 Anatomy, Gandhi Medical College, Hyderabad, IND; 4 Anatomy, All India Institute of Medical Sciences, Bibinagar, Bibinagar, IND; 5 Health Promotion & Health Education, Umm Al-Qura University, Makkah, SAU; 6 Physical Education, Moscow Polytechnic University, Moscow, RUS; 7 Pharmaceutics and Pharmaceutical Biotechnology, Surya School of Pharmacy, Surya Group of Educational Institutions, Villupuram, IND

**Keywords:** cancer genetics, oncology, clinical cancer genetics, study of inherited cancer syndromes, cancer genetic testing

## Abstract

Cancer genetic testing is a revolutionary medical approach that involves the assessment of genetic markers in asymptomatic individuals to predict their future susceptibility to cancer. This paradigm shift in early detection and intervention has the potential to profoundly alter our strategies for cancer prevention and treatment. One pivotal area where genetic testing can have a significant impact is among families with a hereditary predisposition to cancer. Recent research has seen a surge in the exploration of how individuals perceive their cancer risk within the realm of cancer genetics. This proactive approach to genetic testing allows healthcare professionals to identify family members who may carry the same cancer-related genetic mutations, empowering them to make informed decisions regarding their healthcare and cancer risk management. Genetic testing for cancer-related disorders has significantly improved in accuracy and affordability, potentially revolutionizing monitoring and treatment methods. The expanding knowledge of genetic mutations associated with cancer susceptibility has driven significant progress in cancer therapy. Identifying numerous major cancer susceptibility genes has propelled predictive genetic testing, providing individuals with valuable insights into their genetic predisposition to cancer. While perceived risk plays a vital role in genetic counseling, it is equally essential to offer comprehensive information about the advantages and potential risks associated with genetic testing. Ensuring that individuals have a clear understanding of the benefits and potential drawbacks of genetic testing is imperative for making informed healthcare decisions. In our comprehensive review, researchers explored several critical aspects of genetic testing in the context of cancer, including awareness and knowledge, the communication of cancer genetic risk, genetic testing for inherited cancer syndromes, and the challenges and limitations linked to genetic testing. Through this examination, we aim to illuminate the transformative potential of genetic testing in cancer prevention and treatment.

The article "Genetic Testing for Successful Cancer Treatment" was retracted in 2025. Reason: concerns about the authorship.

## Introduction and background

Clinical cancer genetics has emerged as an integral component of cancer patient care. Syndromes such as multiple endocrine neoplasia type 2, von Hippel-Lindau disease, and familial adenomatous polyposis exemplify cases in which genetic testing aimed at identifying at-risk family members is considered the gold standard of care [1]. The sensitivity and affordability of genetic testing for these syndromes have transformative potential in medical management. Our understanding of genetic mutations linked to cancer susceptibility has expanded exponentially, driven by the discovery of numerous major cancer susceptibility genes, thereby advancing predictive genetic testing significantly [2]. Consequently, individuals carrying these mutations can be identified well before cancer onset, allowing them to proactively embrace personalized risk-management strategies to mitigate their cancer risk. This paradigm shift in early detection and intervention holds the promise of revolutionizing cancer prevention and treatment, ushering society into a transformative healthcare era where personalized approaches have the potential to save numerous lives. Predictive genetic testing represents a transformative medical approach that employs genetic testing on seemingly healthy individuals to predict their future disease risks [3]. These tests, distinct from traditional diagnostic tests, are geared toward identifying potential health issues before symptoms manifest to enable early detection of at-risk individuals. This approach, underpinned by precise screening, vigilant monitoring, and tailored preventive measures, can potentially reduce illness and death rates [4]. The utilization of genetic data in this manner has inaugurated a new epoch of personalized healthcare, fostering hope for healthier and extended lives for many. Typically, the process of genetic testing to assess cancer risk commences with an individual who has been diagnosed with cancer within the family. Once a specific genetic mutation associated with an elevated cancer risk is identified in this affected family member, it paves the way for screening other relatives. This proactive approach facilitates the identification of family members who may also carry the same mutation, enabling them to make informed decisions about their healthcare and cancer risk management [5]. Consequently, this cascade genetic testing strategy can significantly enhance early detection and prevention efforts within families characterized by hereditary cancer predisposition. Established genetic counseling and testing protocols are pivotal in evaluating and addressing cancer risk, with a primary focus on effective risk communication to comprehensively inform individuals and their families about their unique susceptibility to cancer [6]. Genetic counselors adhere to these guidelines, imparting essential knowledge regarding personal cancer risk and its familial implications. This holistic approach ensures that inherited cancer risk is comprehended and deliberated within the context of family dynamics, thereby facilitating informed decisions concerning genetic testing [7,8]. Furthermore, these protocols underscore the importance of open and transparent dialogues between healthcare professionals and patients, fostering a collaborative and supportive environment that empowers individuals to make informed choices about their genetic health. Cancer genetic counseling and testing prove particularly advantageous in syndromes such as hereditary breast cancer syndromes, hereditary nonpolyposis colorectal cancer syndrome, Peutz-Jeghers syndrome, and juvenile polyposis [9]. However, certain hereditary cancer syndromes lack available or medically impactful testing, such as Li-Fraumeni syndrome and hereditary malignant melanoma [10]. Comprehensive medical care necessitates the identification of families with probable hereditary cancer susceptibility syndrome, warranting referral to cancer genetics professionals.

The article "Genetic Testing for Successful Cancer Treatment" was retracted in 2025. Reason: concerns about the authorship.

## Review

Awareness and knowledge of genetic testing

Genetic testing for disease susceptibility, particularly in conditions such as cancer, has garnered considerable optimism within public perception [11]. This sentiment was echoed in a Dutch poll where 64% of respondents believed in the potential benefits of genetic testing. However, alongside this optimism, there exists a noteworthy apprehension among the public regarding the potential misuse of genetic test results, which could lead to discriminatory attitudes toward individuals with genetic predispositions [12]. Despite the promising prospects of genetic testing in assessing cancer risk, several ethnic minority communities in both Europe and the United States have encountered significant disparities in their access to genetic services and representation in research endeavors [13]. An earlier assessment focused on the barriers faced by ethnic minorities, such as South Asian, White Irish, and African communities, in their pursuit of cancer genetic services. This evaluation identified multifaceted challenges, including limited awareness and knowledge of available genetic testing services, language barriers, the stigma associated with being at risk, fatalistic attitudes toward cancer, the anticipation of negative emotional responses, uncertainty regarding the information provided, and a prevailing mistrust regarding the use of data [14]. Insufficient comprehension of the significance of genetics concerning cancer, BRCA mutations, and genetic testing has also been observed in various studies involving populations such as Chinese Australians, Hispanics, and African Americans. Generational disparities in awareness, knowledge, and beliefs, especially pronounced in Chinese Australian and Hispanic populations, may have contributed to reluctance toward genetic testing for cancer susceptibility among older generations. Some Chinese Australian participants noted that traditionalists and older generations tended to attribute diseases to misfortune or past transgressions rather than considering the inheritance of mutated genes [15]. Inadequate familiarity with hereditary cancer and limited exposure to genetic testing may act as deterrents for individuals considering such testing. Additionally, differing interpretations of the term "close relatives" may impede the accurate assessment of cancer risk within Chinese Australian groups. Similarly, the strong emphasis on family ties among Hispanic women may influence their attitudes toward genetic testing and their perception of cancer risk. These varied perspectives underscore the importance of identifying and addressing obstacles specific to each ethnic group, necessitating tailored solutions to mitigate these issues. Privacy concerns and the potential for discrimination by disclosing genetic data to third parties, such as insurers and employers, constitute significant drawbacks of genetic testing. The fear that employers or health insurers might gain access to such data has dissuaded many Americans from undergoing genetic testing, with some individuals even forgoing medical care or insurance claims to protect their employment opportunities (Figure 1). Surveys conducted in Canada and Europe have uncovered analogous apprehensions about privacy within the context of genetic testing [16].

The article "Genetic Testing for Successful Cancer Treatment" was retracted in 2025. Reason: concerns about the authorship.

**Figure 1:** Infographics representation of cancer genetics Image credit: Prof. Muthu Prasanna (corresponding author)

Risk of communication of cancer genetic testing

Risk communication is a pivotal component of genetic counseling and testing, and an array of research findings has highlighted its intricacies. Even individuals with a low to moderate risk of developing cancer tend to overestimate their risk, a phenomenon exacerbated by a family history of the disease. Widespread awareness of the potential risks associated with genetic testing is limited, and decision-making regarding genetic testing often hinges on inflated perceptions of cancer risk, eclipsing the actual hazards intrinsic to the testing process [17]. Traditional counseling and educational approaches often struggle to influence individuals' beliefs about their cancer risk, as the processing of risk information is significantly molded by psychological discomfort and coping mechanisms, substantially impacting decisions related to genetic testing. Family dynamics play a crucial role in influencing risk awareness, the decision-making process concerning genetic testing, and ultimate outcomes. Effective pretest counseling mandates a comprehensive exposition of the potential hazards associated with genetic testing [18]. Posttest counseling assumes a central role, encompassing the interpretation of genetic test results, the assessment of individual and family-specific cancer risks, and the presentation of viable risk management options. For participants in genetic counseling programs, a profound comprehension of the complexities of risk is indispensable, as it fundamentally shapes decisions concerning genetic testing and risk management. Unsurprisingly, the realm of cancer genetics has recently witnessed a surge in research on risk perception and communication techniques. It is noteworthy that inherited mutations, in contrast to modifiable cancer risk factors such as lifestyle choices, remain beyond an individual's control. [19] Although the effectiveness of strategies for individuals with these mutations remains unverified, informing carriers of cancer-predisposing mutations about cancer screening and risk reduction options is indispensable. Family knowledge of a relative's test results not only elucidates one's risk status but also significantly impacts psychological well-being. A recurring discovery is that individuals frequently overestimate their cancer risk despite being unaware of all the risk factors and genetic predispositions. Interestingly, gender differences in perceived risk persist despite the gender-neutral nature of genetic inheritance. Genetic counseling may not substantially alter the perceptions of cancer risk or deter interest in testing, even for those with a lower perceived risk threshold. It is essential to provide comprehensive information on the benefits and risks of testing, given that perceived risk is a critical aspect of genetic counseling. Importantly, it has been observed that the adoption of genetic testing is more influenced by perceived risk than actual risk, particularly in the context of colon cancer [20]. Inherited risk is inherently familial, underscoring the importance of effective family risk communication in guiding decisions and shaping testing outcomes. Emotions significantly impact individuals' processing of risk-related information, particularly when faced with a serious health hazard. The challenge of conveying accurate risk information for genetic testing to educators and counselors necessitates exploring new communication techniques. Urgent research is needed to further enhance the methodology and communication materials for genetic testing in the future [21]. This research should extend beyond examining intentions and delving into the actual testing choices and outcomes. While current risk assessments often focus on lifetime cancer risks, a shift toward immediate relevance assessments may prove more useful in genetic testing. Reconsidering counseling strategies is prudent, as genetic counseling requires a substantial time commitment. In the contemporary landscape, transitioning to an approach that prioritizes minimal pretest counseling followed by comprehensive counseling for individuals testing positive for harmful mutations may be more effective [22].

The article "Genetic Testing for Successful Cancer Treatment" was retracted in 2025. Reason: concerns about the authorship.

Genetic testing for inherited cancer syndromes

Multiple endocrine neoplasia (MEN) encompasses a constellation of hereditary cancer disorders, some of which include thyroid tumors. Medullary thyroid carcinoma (MTC), a relatively rare malignancy accounting for 10%-15% of thyroid cancer cases, is diagnosed in about 25% of MEN cases. The most prevalent MEN subtype is MEN2A, where nearly all cases (99%) exhibit MTC, along with pheochromocytoma and hyperparathyroidism. The expression of MEN 2 shows dominant inheritance, and intriguingly, research from the International RET Mutation Consortium reveals germline RET mutations in 92% of MEN 2 cases [23]. The M918T mutation within exon 16 represents approximately 95% of MEN 2B mutations, while the A883F mutation in exon 15 is detected in 5% of cases. In the past, preemptive thyroid removal and continuous monitoring for pheochromocytoma and hyperparathyroidism were necessary, with genetic testing recommended before preventative surgery or by age six. After six years of age, individuals with RET mutations should undergo annual testing for pheochromocytoma and hyperparathyroidism, and they may be considered for thyroidectomy. Von Hippel-Lindau syndrome (VHL) is characterized by renal cell carcinoma, pheochromocytoma, and hemangioblastomas as its hallmark features. The risk of renal cell carcinoma and retinal/cerebellar hemangioblastoma escalates by 70% because of age-dependent VHL penetrance. VHL tumor suppressor gene mutations are associated with autosomal dominant inheritance. Cowden syndrome (CS), connected to PTEN gene mutations, is linked to an increased risk of breast, thyroid, and endometrial cancer. The relationship between CS and the PTEN gene is evident. Li-Fraumeni syndrome (LFS) is an uncommon autosomal dominant cancer syndrome that manifests with various tumor types and is connected to TP53 mutations. Hereditary nonpolyposis colon cancer syndrome (HNPCC) results from mutations in DNA mismatch repair genes, such as MLH1, MSH2, MSH6, and PMS2. This condition elevates the risk of colorectal and endometrial cancer and, in rare cases, is associated with colorectal cancer and brain tumors in Turcot syndrome. Peutz-Jeghers syndrome (PJS) is identified by LKB1/STK11 mutations and distinctive hyperpigmented macules. CDKN2A mutations are frequently linked to hereditary melanoma, whether or not dysplastic nevi are present in (Table 1) [24].

The article "Genetic Testing for Successful Cancer Treatment" was retracted in 2025. Reason: concerns about the authorship.

**Table 1:** Hereditary cancer syndromes Table Credits: [25]

Syndrome	Associated genes	Predominant tumor types or abnormalities
Hereditary breast and ovarian cancer	BRCA1, BRCA2	Breast carcinomas, ovarian carcinomas
Carney complex	PRKAR1A	Skin pigment abnormalities, endocrine tumors, schwannomas
Cowden syndrome	PTEN	Breast carcinomas, thyroid carcinomas, endometrial carcinomas
Familial adenomatous polyposis	APC	Adenomatous polyps of the colon/rectum, gastrointestinal cancers, papillary thyroid carcinomas
Familial melanoma	CDKN2A, CDK4	Cutaneous malignant melanoma, pancreatic cancers
Hereditary papillary renal carcinoma	MET	Papillary renal-cell carcinomas
Hereditary non-polyposis colorectal cancer	MSH2, MSH6, MLH1, PMS1, PMS2	Colorectal and endometrial adenocarcinomas
Hereditary diffuse gastric cancer	CDH1	Diffuse adenocarcinomas of the stomach wall
Juvenile polyposis coli	MADH4	Multiple juvenile polyps in the gastrointestinal tract, colorectal and gastrointestinal malignancies
Li–Fraumeni syndrome	TP53	Breast cancers, soft-tissue sarcomas, brain tumors, adrenocortical tumors, leukemia
Multiple endocrine neoplasia type 1	MEN1	Primary hyperparathyroidism, pancreatic islet-cell tumors, anterior pituitary tumors
Multiple endocrine neoplasia type 2	RET	Medullary thyroid carcinomas, pheochromocytomas, mucosal neuromas
Nevoid basal-cell carcinoma syndrome	PTCH	Basal-cell carcinomas
Neurofibromatosis type 1	NF1	Neurofibrosarcomas, astrocytomas, melanomas, rhabdomyosarcomas, chronic myeloid leukemia
Neurofibromatosis type 2	NF2	Bilateral vestibular schwannomas, meningiomas, spinal tumors, skin tumors
Peutz–Jeghers syndrome	STK11	Gastrointestinal-tract carcinomas, breast carcinomas, testicular cancers, gynecological malignancies
Pheochromocytoma	SDHB, SDHC, SDHD	Pheochromocytomas, glomus tumors
Retinoblastoma	RB	Pediatric retinal tumors
Tuberous sclerosis complex	TSC1, TSC2	Multiple hamartomas, renal-cell carcinoma, astrocytomas
von Hippel–Lindau disease	VHL	Renal-cell carcinomas, retinal and central nervous system haemangioblastomas, pheochromocytomas

Genetic testing for multiple endocrine neoplasia

Mutations within the RET proto-oncogene lead to the rare disorder termed multiple endocrine neoplasia type 2. Individuals affected by this condition face a significantly heightened risk of developing medullary thyroid cancer unless they undergo a preventive surgical intervention involving the removal of the thyroid gland, known as prophylactic thyroidectomy [26]. Through five comparative studies involving pediatric patients diagnosed with multiple endocrine neoplasia type 2, those who underwent thyroidectomy demonstrated compelling evidence of reduced cancer-related mortality compared to those who did not undergo thyroidectomy. The application of predictive genetic testing facilitates the identification of individuals who stand to benefit from such surgical interventions. MEN2, a syndrome marked by the occurrence of medullary thyroid cancer (MTC), unilateral or bilateral pheochromocytoma, and hyperparathyroidism, encompasses various manifestations. Within the spectrum of multiple endocrine neoplasia type 2 (MEN2), familial medullary thyroid carcinoma (FMTC) emerges as a distinct subtype, where individuals manifest solely with MTC without additional symptoms indicative of MEN2. The identification of mutations in the RET proto-oncogene, both in MEN2 and FMTC, provides a precise method for recognizing carriers of the gene. Over the past three decades, persistent efforts have been directed toward mitigating the impact of inherited medullary thyroid cancer as a significant contributor to morbidity and mortality. The revelation of mutations in the RET proto-oncogene in MEN2 presents a unique opportunity to investigate whether prophylactic thyroidectomy can forestall the onset of illness and mortality attributed to hereditary MTC. MEN2A, comprising three distinct variations, includes a subtype characterized by the presence of Hirschsprung disease. In this genetic variant, children exhibit symptoms of Hirschsprung disease at a young age. Although occurrences of this variant in discrete family groups are infrequent, with fewer documented cases, the presence of Hirschsprung disease in individuals within MEN2A family groups suggests that the full spectrum of manifestations may not be comprehensively documented [27]. The condition affects a small number of families, often about 20-30, and it is characterized by the simultaneous presence of MEN2A and cutaneous lichen amyloidosis. People with this genotype exclusively get itchy skin symptoms of amyloid on their upper back. Additionally, FMTC, which is a specific kind of multiple endocrine neoplasia kind 2A (MEN2A), is distinguished by the presence of MTC but does not exhibit the other symptoms often associated with MEN2 [28]. MEN2B, a subtype of MEN2, is comparatively less prevalent than MEN2A, but it still manifests with distinctive characteristics within this condition. Children with this variation frequently demonstrate a reduced ratio between their upper and lower body proportions. While resembling Marfan syndrome, MEN2B lacks the associated abnormalities in the vascular system or eyes. Early identification of MTC in MEN2B is imperative because of the propensity for metastases within the first year of life. Managing MTC poses challenges owing to the frequent oversight of its phenotype. Lymph node metastasis typically occurs within the first 10 years, but distant metastasis becomes more likely to occur. The discovery of RET proto-oncogene mutations in 1993 was a significant breakthrough in the treatment of hereditary MTC or multiple endocrine neoplasia type 2 (MEN2) [29]. About 80% of reported MEN2 mutations can be attributed to the mutation of codon 634, featuring a substitution of a single cysteine with arginine in over half of MEN2A families. The codons 883, 918, or 922 have an effect on 3-5% of all RET mutations. Genetic information enables the evaluation of pheochromocytoma risk, particularly in individuals with RET mutations on specific codons. Individuals with codon 768 and V804M mutations have a low probability of developing pheochromocytoma, which is probably linked to MTC. A comprehensive evaluation of patients displaying apparently random MTC is likely to reveal underlying inherited RET mutations, potentially aiding in identifying other unaware gene carriers. Performing genetic testing multiple times mitigates errors stemming from Taq polymerase-induced alterations or sample contamination. While accredited laboratories employ measures to minimize cross-contamination. Using genetic testing in the clinical management of MEN2 and associated endocrine tumor syndromes has significantly improved the accuracy of syndrome diagnosis, significantly improving the outlook for individuals with these conditions to lead fulfilling and typical lives.

The article "Genetic Testing for Successful Cancer Treatment" was retracted in 2025. Reason: concerns about the authorship.

Genetic testing for hemochromatosis

Hemochromatosis genetic testing is an essential diagnostic technique that identifies inherited variables affecting iron metabolism. Preventive measures to avoid iron overload may be facilitated by identifying genetic predisposition by detecting mutations in the HFE gene. Through this individualized strategy, people may take charge of their health and reduce the risk of consequences related to hemochromatosis. Hemochromatosis is a relatively uncommon disorder characterized by the abnormal accumulation of iron in tissues, resulting in the development of diabetes, cirrhosis, cardiovascular disease, arthritis, and gonadal dysfunction [30]. Phlebotomy emerges as a straightforward and effective preventive therapy, and the application of predictive genetic testing proves valuable in raising suspicion about this occasionally elusive diagnosis. Unlike the evaluation for multiple endocrine neoplasia type 2, the utility of testing for hemochromatosis is comparatively lower because of its limited predictive value. The excessive buildup of iron is rooted in a genetic predisposition. Other factors, such as gender, dietary choices, and exposure to liver toxins like alcohol also play a role in the development of clinically severe iron overload. The penetrance of the hemochromatosis genotype refers to the proportion of persons with the genetic predisposition who would actually develop the associated clinical disease., is relatively low. Hereditary hemochromatosis (HH) represents a prevalent genetic disorder affecting approximately 300 individuals of northern European ancestry. It significantly influences iron management and, if left untreated, can result in liver cirrhosis, hepatocellular carcinoma, diabetes mellitus, cardiomyopathy, and other illnesses linked to early death. Presently, three distinct genetic subgroups of hemochromatosis have been identified. Type 2 HH, genetically linked to chromosome 1q (HFE2), primarily affects individuals with juvenile hemochromatosis, and it is distinct from the more common form occurring later in life. Hoff et al. identified a mutation in the transferrin receptor-2 (TFR2) gene at codon 250, where tyrosine is replaced with a stop signal associated with Type 3 [31]. Subsequent research confirmed this mutation's location at chromosome 7q22 (HFE3). Another report identified a point mutation in the iron response element motif of H-ferritin mRNA in a Japanese family, enhancing cellular iron uptake. Nevertheless, type 1 HH remains the most prevalent variant [32].

Genetic testing in colorectal cancer

Proactive genetic testing proves advantageous when addressing instances characterized by a pronounced familial medical history of a specific ailment. This typically involves three or more affected relatives, with at least one diagnosis occurring before the age of 50, particularly when suggestive of hereditary non-polyposis colon cancer. The implementation of routine colonoscopic surveillance in these individuals demonstrates a notable reduction, specifically a 62% decrease, in the incidence of colorectal cancer compared to those who do not undergo such monitoring [33]. Colorectal cancer persists as the third most common type of cancer in both males and women in the United States. Approximately 33% of CRC cases are identified in individuals with a familial history of the condition. Numerous genes have been associated with hereditary cancer syndromes characterized by a single gene anomaly, many of which elevate the susceptibility not only to colorectal cancer but also to other tumor types. The characteristics of colorectal polyps include their number, size, histology, and location [34]. Endoscopic procedures prove effective in reducing CRC risk by removing those polyps, which generally arise because of somatic genetic events affecting critical cellular functions such as proliferation, migration, apoptosis, and DNA repair. As individuals age, the occurrence of colorectal polyps and CRC escalates. Screening for colorectal neoplasia stands as a successful strategy to mitigate CRC risk, with guidelines recommending initiation at the age of 50. Moreover, individuals with an average risk should undergo this procedure, while those with an increased risk may consider it at an earlier age. The significance of family history is crucial in predicting the risk of colorectal cancer (CRC), as the risk increases in proportion to the number of relatives affected. Considering that adenomatous polyps are the main antecedents to most colorectal cancers (CRCs), the primary approach to reducing the risk in patients with adenomatous polyposis is to remove as many polyps as possible. The standard treatment for individuals with identifiable polyposis features usually consists of surgical intervention, which can be accomplished through colectomy with ileocecal anastomosis or proctocolectomy with ileal J-pouch-anal anastomosis. Individuals diagnosed with attenuated adenomatous polyposis may choose vigilant monitoring through endoscopic polypectomies as an alternative to surgical intervention. Genetic testing plays a pivotal role in shaping the clinical management of closely related individuals, enabling the identification of hereditary mutations in affected individuals to establish specific syndrome diagnoses. This, in turn, facilitates the extension of genetic testing to at-risk family members. The Cancer Genome Atlas has uncovered notable genetic heterogeneity within CRCs. Despite more than 80% of CRCs manifesting somatic mutations in the APC gene, a distinct subset exhibits unique gene mutation profiles, and over 13% lack APC mutations [35]. While genetic testing is valuable for confirming syndromic diagnoses in non-adenomatous polyposis cases, its clinical utility is often limited. CRC screening has proven effective in mitigating morbidity and mortality linked to CRC. Ideally, aligning CRC screening with risk levels would be optimal, but the challenge lies in accurately identifying individuals who would benefit most from specialized surveillance. Traditional reliance on clinical history as the cornerstone for assessing CRC risk is complicated by variations in clinical characteristics and disease manifestation likelihood. Advanced parallel next-generation sequencing techniques, encompassing whole exome or genome analyses, hold promise for unveiling new genes or gene combinations contributing to genetic susceptibility. While colorectal cancer screening is a vital means for reducing the disease's negative effects on health, there is still work to be done in terms of accuracy. Although proper risk evaluation is complex, it is a desirable objective for customizing screening to individual risk levels. With the field of sophisticated DNA sequencing tools developing, there is optimism that additional aspects of genetic vulnerability may be found, opening the door for further focused and successful colorectal cancer prevention efforts.

The article "Genetic Testing for Successful Cancer Treatment" was retracted in 2025. Reason: concerns about the authorship.

Genetic testing in breast and ovarian cancer

Genetic testing that can anticipate the likelihood of developing breast and ovarian cancer, as well as hereditary non-polyposis colon cancer, holds considerable promise in identifying individuals at heightened risk for these diseases. Individuals carrying genetic alterations in the BRCA1 or BRCA2 genes face varied potential outcomes, including the risk of developing cancer. The options are breast cancer, ovarian cancer, both cancers, or neither. Approximations of penetrance for breast cancer range from 36% to 85%, and for ovarian cancer, the range is 10% to 44%, with significant age-related variability in cancer occurrence [36]. These uncertainties stem from diverse factors, including environmental influences, evolving genetic factors, individual-specific mutations in women, and stochastic events. Moreover, the efficacy of predictive genetic testing is further constrained by the characteristics of existing surveillance and preventive measures. Recommendations for individuals with the BRCA1 or BRCA2 gene include commencing mammography between the ages of 25 and 35, although the effectiveness of early monitoring remains uncertain. Tamoxifen chemoprevention demonstrates potential in mitigating the likelihood of breast cancer, while there is contradictory evidence [37]. Oral contraceptives can reduce the chances of getting ovarian cancer; however, simultaneously, they may increase the risk of acquiring breast cancer. Prophylactic oophorectomy and mastectomy are effective choices for certain women, showing effectiveness in decreasing the risk of cancer. Females commonly experience the onset of breast and ovarian tumors, constituting prevalent cancer types. The increasing recognition of genetic predisposition as a significant risk factor in the occurrence of these cancers emphasizes the importance of BRCA1 and BRCA2 genes in hereditary breast and ovarian cancer. Recent advancements in molecular techniques, including next-generation sequencing, have revealed a multitude of new genes linked to the vulnerability to breast and/or ovarian cancer. Each of these genes has different estimates of how likely they are to cause the disease. Genes with high penetrance, such as TP53, PTEN, STK11, and CDH1, significantly increase the likelihood of developing breast and ovarian cancers. Furthermore, PALB2, BRIP1, ATM, CHEK2, BARD1, NBN, NF1, RAD51C, RAD51D, and mismatch repair genes are the most important. Beyond breast and ovarian cancers, an amalgamation of environmental and genetic variables contributes to their manifestation [38]. Familial clustering is evident in approximately 10-30% of cases, with hereditary cases accounting for an estimated 5-10% linked to specific genetic mutations. The BRCA1 gene, situated on chromosome 17q21.31, produces a nuclear protein that plays a role in repairing DNA, regulating the cell cycle, and maintaining the stability of the genome. BRCA1 functions as a tumor suppressor by working with other suppressors, sensors, and transducers to create a complex called the BRCA1-associated genome surveillance complex (BASC). While BRCA1 and BRCA2 are well-recognized breast and ovarian cancer susceptibility genes, emerging data from next-generation sequencing highlight novel genes contributing to predisposition. Despite this, routine testing beyond BRCA1/2 is infrequent because of limited risk information and the absence of monitoring programs. Notably, genes like TP53, PTEN, STK11, CDH1, and PALB2, although with varying penetrance, demand inclusion in comprehensive gene panels for identifying individuals susceptible to breast or ovarian cancer. Next-generation sequencing has uncovered unexpected links between genetic reasons predisposing to breast and ovarian cancer and gastrointestinal tumors. This intersection of cancer genetic predisposition and precision medicine is exemplified by PARP inhibitors as potential therapies for individuals carrying pathogenic or likely pathogenic variants in BRCA1/2 genes, initially effective in treating ovarian cancer and subsequently in breast, prostate, and pancreatic cancers [39]. Genetic testing can also be used to identify circulating tumor DNA (ctDNA), a biomarker for breast cancer. ctDNA is a small amount of tumor DNA that can be found in the blood. Genetic testing can detect specific mutations in ctDNA that are associated with breast cancer. This information can be used to diagnose breast cancer, determine the type and stage of cancer, and guide treatment decisions [40]. Significant associations among genetic susceptibility for ovarian, gastrointestinal, and breast cancers have been revealed by next-generation sequencing. PARP inhibitors are a prime example of the intersection of personalized medicine and genetic knowledge since they have been shown to be effective against a variety of cancer types. Genetic testing becomes an essential tool for breast cancer options for therapy, providing accurate diagnosis and identifying circulating tumor DNA.

The article "Genetic Testing for Successful Cancer Treatment" was retracted in 2025. Reason: concerns about the authorship.

Psychological concern for GT

Despite potential psychological and societal concerns, empirical data from controlled outcome studies conducted in the United States, Europe, and Australia have not revealed significant or widespread negative psychological effects associated with genetic testing among high-risk individuals [41]. Although the current outcome data provide grounds for optimism regarding the psychological impacts of receiving cancer-susceptibility test results, it is crucial to acknowledge specific limitations or conditions. Genetic testing may give rise to subtle consequences, including anxiety, apprehensions about cancer, familial tensions, and complexities in medical decision-making. These effects have been documented in individuals testing positive for particular genetic conditions, and, in some instances, they can exert a substantial adverse influence on the quality of life for these individuals. Moreover, while the majority of individuals appear to exhibit positive psychological responses to genetic testing, there exists a distinct minority who may encounter negative psychological implications, as previously mentioned [42]. Hereditary cancer risk counseling encompasses the identification of families predisposed to hereditary cancer syndromes, with the primary aim of mitigating the incidence of cancer-related morbidity and mortality. This often involves advising individuals from families with known hereditary cancer syndromes to undergo more frequent and earlier screening alongside other risk-reduction strategies. Preceding genetic testing, it is recommended to undergo counseling regarding the hereditary cancer risk, facilitating informed decision-making by the patient. Typically, initial testing is conducted on a family member with a personal history of the specific cancer type under evaluation. Within the family, individuals with a past occurrence of the particular inherited cancer are designated as "affected family members," while those lacking a personal history of the disease are termed "unaffected family members." Moreover, individuals testing positive for a mutation are commonly referred to as carriers. Despite numerous studies exploring potential rises in distress, limited attention has been given to evaluating the positive psychological analysis of genetic counseling and test reporting and their possible advantages. Gage et al. conducted a comprehensive research study that uncovered multiple ways, wherein cancer genetic counseling and a positive test result can impact the self-perception of those at high risk for cancer [43]. The study sought to evaluate the influence of counseling and testing on self-perception by conducting individual interviews and focus groups with both affected and unaffected individuals. There is a growing belief that predictive genetic testing for hereditary cancer risk should be acknowledged as an essential part of an ongoing effort to address the psychological and behavioral aspects of familial cancer risk. Genetic counseling and testing play a crucial role in effectively managing the risk of inherited cancer across various cancer syndromes. Hereditary cancer risk counseling and testing are essential components in an ongoing practice under this paradigm. Hereditary cancer risk counseling and testing have a significant impact on the extent to which individuals follow screening regimens and engage in other actions that reduce their risk, such as undergoing preventative surgery. In cases such as hereditary melanoma, they can assume a critical role in advocating primary prevention measures, notably reducing exposure to ultraviolet radiation (UVR) [44]. These findings underscore the multifaceted contributions of genetic cancer risk counseling and testing, not only to early detection efforts with potentially life-saving implications but also to proactive preventive initiatives. Existing research generally refutes the notion that cancer genetic testing precipitates enduring psychological distress. Nevertheless, there is a growing acknowledgment that diverse patterns of outcomes may exist, and certain patient subsets may be susceptible to heightened levels of sadness and/or anxiety. Proactively identifying individuals predisposed to such responses enables targeted and effective intervention efforts. Expanding beyond considerations of depression, anxiety, and cancer-related concerns, investigations into various psychological outcomes reveal that patients often encounter both advantages and drawbacks associated with inherited risk counseling and testing. Qualitative data from structured interviews and open-ended survey questions indicate substantial benefits, some of which may not be entirely captured by standardized measurements. It is imperative to comprehend the intricate interplay between positive and negative consequences resulting from positive test results, subsequent screening behaviors, and the adoption of recommended health strategies to mitigate risk.

The article "Genetic Testing for Successful Cancer Treatment" was retracted in 2025. Reason: concerns about the authorship.

Challenges and limitations of genetic testing

In the realm of genetic testing, comparative genetic testing primarily illuminates the potential for future health conditions, but it does not definitively determine their manifestation. The level of uncertainty associated with these findings remains substantial, even in cases where the identified risk is notably high, such as a positive test for Huntington's disease. This unpredictability extends to not only whether the specific ailment will indeed develop but also to the timing and severity of its onset. Moreover, the inherent uncertainty is amplified in the context of predictive genetic testing because of the typically unproven nature of risk-reduction treatments [45]. Recommendations often hinge on anticipated advantages rather than empirically established outcomes. Notably, predictive genetic testing diverges from traditional diagnostic tests in its immediate impact on not only the individual but also their family members. The motivation for undergoing such testing often arises from concerns about the health of relatives. However, the utility of predictive genetic testing can diminish when medical advances render previously menacing conditions, such as breast or colon cancer, increasingly treatable through less-invasive methods. Additionally, the widespread availability of efficient screening techniques across the general population may diminish the necessity for comprehensive predictive genetic testing [46]. Conversely, the appeal of predictive genetic testing rises as the costs associated with screening increase, particularly when more expensive yet superior techniques, like magnetic resonance imaging, outweigh relatively affordable alternatives such as mammography. Individuals' suitability for predictive genetic testing is significantly influenced by their personal experiences and family medical history. Various factors can either enhance or diminish the utility of such testing. Conditions characterized by high morbidity and mortality rates, therapies that are effective but not curative, and genetic testing with a high predictive value (high penetrance) are associated with increased utility. Conversely, diseases with lower morbidity and mortality rates, treatments that are both effective and well-tolerated, and genetic tests with lower predictive accuracy (low penetrance) tend to reduce utility. The complexity and cost of screening techniques further influence the utility, with more expensive and cumbersome methods diminishing it, while affordable and efficient approaches enhance it. The value of predictive genetic testing is also affected by the affordability and consequences of preventative actions, with expensive or detrimental measures diminishing its value, while straightforward, effective, and widely accepted preventive measures, such as vaccination, can enhance the overall usefulness of predictive genetic testing. Interpreting the implications of positive or negative test results can be a challenging endeavor, as depicted. Figure 2 illustrates the level of use for different disorders based on their current clinical testing usefulness ranking. The following disorders are addressed below: from the most beneficial cases for testing to the least beneficial ones, testing is least effective or potentially detrimental for situations where its benefits are limited or outweighed by potential negative consequences.

The article "Genetic Testing for Successful Cancer Treatment" was retracted in 2025. Reason: concerns about the authorship.

**Figure 2:** Utility in predictive genetic testing Image credit: [47]

A negative test result often provides reassurance, particularly when the family's predisposing mutation is already identified. In the realm of cancer genetic testing, with a specific focus on breast cancer, the overarching objectives revolve around enhancing patient and public awareness. Augmenting comprehension is vital to align the burgeoning demand with genuine necessities. The field of genetic testing for cancer is currently undergoing a remarkable transformation, steered by several influential factors. An increasing number of laboratories are now offering cancer genetic testing services, mirroring the surging interest in personalized genetic insights concerning cancer risk [48]. In response to this heightened demand, the introduction of multiple testing panels, each encompassing a distinct array of genes, signifies a dedicated pursuit to comprehensively investigate genetic risk factors. Nonetheless, this expansion brings intricacies into play, as it entails the management and interpretation of additional genes, compounded by the unforeseen genetic revelations that carry clinical implications. Variants of unknown significance (VUSs), representing genetic alterations with poorly understood clinical implications, are being unearthed concurrently. The accumulation of these VUSs augments the complexity of the genetic data that is already at our disposal. This progression indicates a societal inclination toward comprehending genetic makeup and its implications, aligned with the growing public interest in genetic testing. Within this evolving landscape, genetic counseling assumes a broader scope, with genetic counselors adeptly navigating a rapidly expanding genetic terrain, handling both validated results and the uncertainties introduced by the discovery of VUSs. There is also a discernible trend toward proactive identification of risks within larger population groups aimed at enabling early interventions and risk management through genetic marker-based population screening. Evidently, the evolving landscape of cancer genetic testing underscores the imperative need for robust clinical decision support (CDS) mechanisms. Such mechanisms are indispensable for translating intricate genetic data into actionable insights that healthcare professionals can effectively utilize, thereby underscoring the dynamic interplay between cutting-edge genetics and judicious medical decision-making [49].

The article "Genetic Testing for Successful Cancer Treatment" was retracted in 2025. Reason: concerns about the authorship.

## Conclusions

Genetic testing addresses several crucial factors: firstly, it recognizes that a substantial proportion of individuals with a familial history of cancer, even those with relatively low to moderate risk levels, often tend to overestimate their susceptibility to cancer. Secondly, it acknowledges the limited awareness concerning the potential risks associated with genetic testing. Thirdly, it underscores the significant impact of exaggerated perceptions of personal cancer risk on decisions regarding genetic testing, with a relatively lesser influence on risk perceptions. To foster greater involvement of racial and ethnic minority groups in upcoming endeavors related to cancer risk prediction, it is imperative to provide culturally relevant information and implement awareness campaigns aimed at reducing the stigma and reservations associated with cancer. These targeted efforts hold the potential to facilitate increased participation. However, despite the promising medical and emotional benefits associated with genetic testing for cancer risk, numerous barriers hinder its widespread practical implementation. Both patients and healthcare professionals must give due consideration to issues of privacy and the looming specter of genetic discrimination, particularly in the context of affordable health insurance. These considerations are vital in shaping the future landscape of genetic testing for cancer risk assessment.
